This article has been retracted.

# LncRNA LIPE-AS1 Predicts Poor Survival of Cervical Cancer and Promotes Its Proliferation and Migration via Modulating miR-195-5p/MAPK Pathway

**DOI:** 10.3389/fonc.2021.639980

**Published:** 2021-04-09

**Authors:** Jie Zhang, Pinping Jiang, Shoyu Wang, Wenjun Cheng, Shilong Fu

**Affiliations:** ^1^Department of Gynecology, The First Affiliated Hospital of Nanjing Medical University, Nanjing, China; ^2^Department of Gynecology, Nanjing Medical University, Nanjing, China; ^3^Department of Molecular and Cellular Oncology, Nanjing University Medical School, Nanjing, China

**Keywords:** cervical cancer, LIPE-AS1, miR-195-5p, MAP3K8, MAPK signaling pathway

## Abstract

**Aims:** A growing number of studies have unveiled that long non-coding RNA (lncRNA) is conductive to cervical cancer (CC) development. However, the effect of LIPE-AS1 is remained to be studied in CC.

**Main Methods:** Reverse transcription-polymerase chain reaction (RT-PCR) was employed to measure LIPE-AS1 expression in CC tissues and the adjacent normal tissues. Additionally, we conducted gain- and loss-of functional experiments of LIPE-AS1 and adopted CCK8 assay, BrdU assay, and *in vivo* tumor formation experiment to test the proliferation of CC cells (HCC94 and HeLa). Besides, the apoptosis, invasion, and epithelial-mesenchymal transformation (EMT) of CC cells were estimated using flow cytometry, transwell assay, and western blot, respectively. Further, LIPE-AS1 downstream targets were analyzed through bioinformatics, and the binding relationships between LIPE-AS1 and miR-195-5p were verified via dual-luciferase activity experiment and RNA Protein Immunoprecipitation (RIP) assay. Moreover, rescue experiments were conducted to confirm the effects of LIPE-AS1 and miR-195-5p in regulating CC development and the expressions of MAPK signaling pathway related proteins were detected by RT-PCR, western blot, and immunofluorescence.

**Key Findings:** LIPE-AS1 was over-expressed in CC tissues (compared to normal adjacent tissues) and was notably related to tumor volume, distant metastasis. Overexpressing LIPE-AS1 accelerated CC cell proliferation, migration and EMT, inhibited apoptosis; while LIPE-AS1 knockdown had the opposite effects. The mechanism studies confirmed that LIPE-AS1 sponges miR-195-5p as a competitive endogenous RNA (ceRNA), which targets the 3′-untranslated region (3′-UTR) of MAP3K8. LIPE-AS1 promoted the expression of MAP3K8 and enhanced ERK1/2 phosphorylation, which were reversed by miR-195-5p.

**Significance:** LIPE-AS1 regulates CC progression through the miR-195-5p/MAPK signaling pathway, providing new hope for CC diagnosis and treatment.

## Introduction

Cervical cancer (CC), as one prevailing gynecological malignant tumor, ranks second among female malignancies following breast cancer, and even ranks first in some developing countries (1). Despite the employment of advanced radio- and chemo-therapy technologies, the prognosis of CC patients is still unsatisfactory because of regional recurrence and distant metastasis (2). Therefore, a profound study on the molecular mechanism on CC development is instrumental for the early diagnosis and treatment for CC.

In recent decades, the effect of lncRNA on CC occurrence and growth has received accumulating attentions (3). For instance, lncRNA MIR210HG was found to be elevated in CC tissues and related to FIGO staging, metastasis and worse survival of CC patients. In addition, it promoted CC proliferation, invasion, and epithelial-mesenchymal transformation (EMT) by regulating the miR-503-5p/TRAF4 axis (4). Li et al. reported that lncRNA CCAT1 was over-expressed in CC tissues, and CCAT1 knockout restrained CC development via inhibiting cell proliferation, migration, invasion, EMT, and accelerating cell apoptosis (5). On the other side, some lncRNAs, such as lncRNA PTENP1, were reported to inhibit cervical cancer development (6). Therefore, lncRNAs may play different roles in CC. LIPE-AS1 is a newly reported lncRNA found in lung and liver cancer cells, and it was found to be inversely co-regulated upon DNA damage (7). However, the effect and mechanism of LIPE-AS1 in the malignant biological behavior of CC are unclear. Thus, we first determined the LIPE-AS1 level in CC tissues and cells and then studied the relationship of LIPE-AS1 level with the clinic pathological characteristics of CC patients.

MiR-195-5p is a type of low-expressed miR-8 in CC tumors (8). Studies have stated that miR-195-5p up-regulation targets MMP14 to inhibit the TNF signaling pathway, thereby inhibiting CC cell proliferation and invasion (8). What's more, miR-195-5p is reported to restrain CC cell malignant biological behavior by inhibiting ARL2 expression (9). Therefore, miR-195-5p targets a variety of different downstream proteins to inhibit CC development and further exploration of miR-195-5p downstream targeted genes in CC may be of great significance for understanding CC.

Among multiple tumors, mitogen-activated protein kinase kinase kinase 8 (MAP3K8) is closely related to the malignant biological behavior of tumors and promotes the development of melanoma (10), squamous cell carcinoma (11), and other tumors. In the meantime, several miRNAs are found to target MAP3K8. For instance, miR-589-5p binds to the 3′-UTR of MAP3K8 mRNA in HCC and down-regulates MAP3K8 expression, thus down-regulating the stemness characteristics of CD90 CSCs (12). Moreover, miR-144-3p can inhibit the invasion and migration of renal cell carcinoma by targeting MAP3K8 (13). Therefore, the regulation of tumor malignant biological behaviors by miRNA-targeted MAP3K8 may be an important mechanism for the regulation of CC.

Besides, papers have manifested that lncRNAs regulates gene expression by targeting miRNAs as a competing endogenous RNA (ceRNA). For example, FOXD2-AS1 up-regulates HDGF by sponging miR-760, which mediates the tumorigenic effect in CC (14). However, the issues that miR-195-5p sponges lncRNA and the regulatory effect of lncRNA/ miR-195-5p/MAP3K8 axis in CC are still unclear. This paper intends to explore whether LIPE-AS1 regulates CC progression by competitively stimulating miR-195-5p to regulate MAP3K8, thereby regulating the malignant biological behaviors of CC. Allover, the present study provides a comprehensive basis for a more profound understanding of CC pathogenesis and pave the way for new perspectives on its treatment.

## Materials and Methods

### Clinical Tissues Collection

From January 2014 to January 2015, 42 CC patients underwent surgical treatment in the First Affiliated Hospital of Nanjing Medical University were chosen. All the patients were not treated with radiotherapy or chemotherapy before they were diagnosed as CC. All cases were diagnosed as CC pathologically according to the world health organization (WHO) criteria (mainly basing on clinical symptoms, histopathological examination, and imaging examination). Those patients with FIGO Stage I-IIA received surgery treatment, while those patients with over Stage IIB were treated with chemotherapy and radiotherapy. We obtained tumor tissues and matched non-tumor tissues during histopathological examination, which were then immediately frozen in liquid nitrogen. The experiments were conducted strictly under the approval of the ethics committee of the First Affiliated Hospital of Nanjing Medical University, and all patients had written informed consent. We followed up all patients for 3 months to 4 years, with death or loss of follow-up as the endpoint.

### Cell Culture

We purchased normal cervical epithelial cell lines HUCEC and cervical cancer cell lines including Hela, MS751, SiHa, CaSki, C-33A, and HCC94 from American Type Culture Collection (ATCC, Rockville, MD, USA). DMEM-F12 medium supplemented with 10 mmol/L HEPES, 10% fetal bovine serum (FBS, HyClone, Logan, UT, USA) and 1% penicillin-streptomycin solution (Beyotime, Shanghai, China) was used for cell culture. The cells went through incubation at 37°C with saturated humidity of 5% CO_2_. We changed the medium every 2–3 days and passaged the cells every 3–5 days by using 0.25% Trypsin (Sigma, CAS:9002-07-7).

### RNA Isolation and Quantitative RT-PCR

TRIzol (Invitrogen) was taken to extract total RNA, and genomic DNA was removed from the total RNA using deoxyribonuclease I. The reverse transcription reaction was performed according to the operation procedure of Thermo Scientific Revert Aid First Strand cDNA Synthesis Kit reverse transcription kit, and the reaction conditions were as follows: 10 min at 70°C, 5 min on ice, 60 min at 42°C, 5 min at 95°C, 5 min at 0°C. The fluorescence quantitative PCR reaction system was 25 μL mixture containing 500 ng cDNA template, 250 nmol/L upper and lower primers, and 12.5 μL of 2×SYBR Green PCR Master. GAPDH was employed as an endogenous control of the target gene. The primer sequence of each molecule is as follows: LIPE-AS1 primer sequence: forward 5′-ACTCCATACTCTCCCTGGGT-3′, reverse 5′-GCTTCTATGCCTTCCTTCCC-3′; miR-195-5p: forward: 5′-CGGGTTCAGCATCAAATGAGAAAGCA-3′ reverse 5′-CAGCAGGTAGAAAGAGCACAAT-3′; GAPDH: forward: 5′-CTCCTCCTGTTCGACAGTCAGC-3′, reverse: 5′-CCCAATACGACCAAATCCGTT-3′ (Sangon Biotech; China). Bcl2: MQP091236; *IGF1R:* MQP029442; *GNA13:* MQP092485; *CDK6:* MQP028861; *IKBKB:* MQP054170; *CCND1:* MQP026722; *E2F3:* MQP078979; *MAPK8:* MQP076511; *FGF2:* MQP027087; *GNAQ:* MQP027212; *AKT3:* MQP030532; *PIAS2:* MQP074629; *WNT3A:* MQP028531; *CCNE1:* MQP026724; *VEGFA:* MQP024363 (Genecopoeia; USA). The reaction tube was placed into the MX3000P Realtime PCR reaction instrument. The reaction conditions were: 94°C 40 s, 55°C 40 s, 72°C 40 s, 45 cycles, and fluorescence signal monitoring. The relative expression of the gene was represented via the 2^−ΔΔCt^ value. The Ct value represents the amplification cycle number that the PCR product passes when the fluorescence signal of the amplified product reaches a set threshold during the PCR amplification process. ΔΔCt = test sample (Ct target gene-Ct GAPDH) -control group (Ct target gene-Ct GADPH).

### Cell Transfection

The short-hairpin RNA (shRNA) targeting LIPE-AS1 (sh-LIPE-AS1), LIPE-AS1 over-expressing plasmids, miR-195-5p mimics, and inhibitors as well as their negative controls were obtained from Shanghai GenePharma Co., Ltd. (Shanghai, China). HCC94 and Hela cells were seeded in the 24-well plates with 2 × 10^5^ cells each well. Lipofectamine 2000 reagent (Sangon Biotech, Shanghai, China) was applied for cell transfection according to the manufacturers' protocol.

### CCK-8 Experiment

The altered cell proliferation ability of HeLa and HCC94 cells at 24, 48, 72, and 96 h after transfection and co-transfection were examined via CCK8 assay (Beyotime Biotechnology, Shanghai, China). HeLa and HCC94 cells (2 × 10^3)^ were taken from each group and inoculated in 96-well plates. After 24 h of culturing, 10 μL CCK-8 solution was added to each well. After 4 h of incubation, the absorbance value at 450 nm was determined with a microplate reader.

### BrdU Experiment

After stable transfection, the cells in the logarithmic growth phase were used to prepare a single-cell suspension, and they were inoculated into 24-well plates at the rate of 1 × 10^5^ cells per hole. After the cells were adherent to the walls, BrdU (50 μmol/L, Sigma, USA) was added, and the plate was placed in an incubator with 5% CO_2_ at 37°C. When a 48-h continuous cell culture was finished, immunofluorescence staining was conducted to mark the BrdU in the cells and the nucleus was stained by DAPI (Beyotime Biotechnology). Under the microscope, the number of BrdU positive cells were calculated. Cell proliferation rate = number of BrdU positive cells/number of DAPI positive cells, and the mean cell proliferation rate of three fields was taken as the cell proliferation rate.

### Flow Cytometry

Flow cytometry was conducted to detect cell apoptosis. After stable transfection, HCC94 and Hela cells in the logarithmic growth phase were inoculated into 24-well plates (1 × 10^5^ cells per well). Then the cells were collected, and cell apoptosis was determined using Annexin V-FITC Apoptosis detection kit (ThermoFisher, Waltham, MA, USA) and the flow cytometer (BD Biosciences, San Jose, CA, USA).

### Transwell Experiment

Before the transwell assay was conducted, the upper Transwell chamber was coated with 20 μL Matrigel (Thermo Fisher Scientific, MA, USA) at 37°C for 30 min to reconstruct the basement membrane. The cells were resuspended in serum-free medium and 100 μL cell suspension was added into the upper chambers. In the lower chamber, 600 μL of complete culture medium containing 10% fetal bovine serum was added and then the plates were placed in the incubator. Twenty-four hours later, we took out the Transwell chambers and wiped off unmigrated cells in the upper chamber with cotton swabs. The cells in the lower chamber were fixed with methanol for 30 min and stained with crystal violet for 15 min. Finally, the number of cells penetrating the basement membrane was counted from 5 fields under a microscope.

### Western Blot

The tissues or cells were collected and lysed with RIPA lysis solution (Beyotime Biotechnology, Shanghai, China) and the total protein was extracted. Next, the protein (30 μg) underwent sodium dodecyl sulfate-polyacrylamide gel electrophoresis (SDS-PAGE) and then were transferred to polyvinylidene fluoride (PVDF) membranes, sealed with 5% skimmed milk powder, and incubated with primary antibodies at 4°C overnight. On the next morning, the membranes were washed with TBST buffer and incubated with horseradish peroxidase (HRP) -labeled anti-rabbit secondary antibodies (Abcam, ab6721, concentration 1: 1,000, MA, USA) for 1 h at room temperature. After washing the membranes by TBST, ECL was added for brands exposure, and Image-J was applied to analyze OD value. Primary antibodies used in this study were as follows: E-cadherin (Abcam, ab40772, concentration 1: 1,000, MA, USA), Snail (Abcam, ab18203, concentration 1:1,000, MA, USA), Vimentin (Abcam, ab92547, concentration 1: 1,000, MA, USA), MAP3K8 (Abcam, ab137589, concentration 1: 1,000, MA, USA), p-ERK (Abcam, ab214362, concentration 1: 1,000, MA, USA), ERK (Abcam, ab17932, concentration 1: 1,000, MA, USA), GAPDH (Abcam, ab128915, concentration 1: 2,000, MA, USA).

### Dual Luciferase Reporter Gene Assay

All luciferase reporter vectors (LIPE-AS1-WT, LIPE-AS1-MUT, MAP3K8-WT, MAP3K8-MUT) were constructed by Promega (Promega, Madison, WI, USA), among them LIPE-AS1-WT, MAP3K8-WT contained the binding sites with miR-195-5p while LIPE-AS1-MUT and MAP3K8-MUT were mutant for the binding sites with miR-195-5p. HCC94 and Hela cells (4.5 × 10^4^) were inoculated in a 48-well plate and cultured till they were reached 70% confluent. Then the vectors of LIPE-AS1-WT, LIPE-AS1-MUT or MAP3K8-WT, MAP3K8-MUT were co-transfected with miR-195-5p mimics or miR-NC using lipofectamine 2000. Finally, the dual luciferase activities were detected following the manufacturer's operational instructions of dual-luciferase assay system (Promega) 48 h after transfection. All experiments were conducted in triplicate and repeated three times.

### RIP Assay

HeLa and HCC94 cells were collected and the Magna RIPTM RNA-binding protein immunoprecipitation kit (Millipore, Bedford, Massachusetts, USA) was used on transfected cells to perform RIP analysis. Then, we incubated the cells with anti-Ago2 antibody (Millipore) or negative control IgG (Millipore) and examined the enrichments of miR-195-5p and LIPE-AS1 in the lysates by qRT-PCR.

### *In vivo* Tumor Formation Assay

Sixty female nude mice (BALB/c, purchased from the animal center of Wuhan University) were raised in SPF conditions. After stable transfection, HeLa and HCC94 cells were collected and resuspend by PBS. Each nude mouse was injected subcutaneously with 0.2 mL of cell suspension (containing 2.0 × 10^7^ cells). During the next 5 weeks of inoculation, the length and width of nodules were measured weekly to calculate the tumor volume. After 5 weeks, the nude mice were sacrificed, the subcutaneous nodules were taken out, and the size and weight of the nodules were calculated.

### Immunofluorescence Experiment

HeLa and HCC94 cells transfected with NC-miR or miR-195-5p mimics were seeded into 24-well plates (5.0 × 10^5^ cells/well). After 24 h, the cells were fixed in 4% paraformaldehyde for 10 min (at room temperature), permeabilized with 0.05% Triton X-100 and blocked with 5% normal goat serum (Beyotime, Shanghai, China) for 1 h (at room temperature). Next, the cells were incubated with primary antibody of MAP3K8 (Abcam, ab137589, concentration 1: 100, MA, USA) for 18 h at 4°C. Followed by that, the cells were washed three times with PBS, incubated with goat anti-rabbit IgG H&L (Alexa Fluor® 488) (Abcam, ab150077; 1:200; MA, USA) for 2 h at 37°C and stained with DAPI (Beyotime, Shanghai, China) at room temperature for 15 min. For detecting MAP3K8 expression in the tumor tissues, the tumor tissues were fixed in 4% paraformaldehyde and 4-μm sections were also prepared. After being permeabilized with 0.05% Triton X-100, blocked with 5% normal goat serum, the sections were, respectively, incubated with primary antibody of MAP3K8 (Abcam, ab137589, concentration 1: 100, MA, USA) and goat anti-rabbit IgG H&L (Alexa Fluor® 594) (ab150080; 1:200; MA, USA). DAPI (Beyotime, Shanghai, China) was used for staining nucleus. The immunofluorescence signal was observed using a fluorescence microscope (×200, Olympus Company).

### Statistical Analysis

SPSS17.0 statistical software (SPSS Inc., Chicago, IL, USA) was employed for analysis. The measurement data were presented as mean ± standard deviation (x ± s). Multi-group data and two-group data were, respectively, analyzed by univariate ANOVA and the independent sample *t*-test. Pearson's correlation analysis was used for analyzing the relations of miR-195-5p and LIPE-AS1 in CC tissues. *P* < 0.05 has statistically significant.

## Results

### LIPE-AS1 High Expression Is Associated With Poor Prognosis of CC Patients

Aiming at the study of LIPE-AS1 expression in CC and its relationship with pathological features, RT-PCR was utilized to test the level of LIPE-AS1 in CC tissues and cell lines. The results showed that LIPE-AS1 was remarkably up-regulated in CC tissues (Figure 1A). Besides, higher level of LIPE-AS1 was significantly associated with the increasing of FIGO stage (Figure 1B). Through the GEPIA database (http://gepia.cancer-pku.cn/), it was indicated that compared with normal tissues, LIPE-AS1 expression was notably increased in Cervical squamous cell carcinoma and endocervical adenocarcinoma (CESC) (Figure 1C). Moreover, we analyzed the prognosis of CC patients with different levels of LIPE-AS1, the results suggested that higher level of LIPE-AS1 was related with lymph node metastasis of CC patients (Table 1). What's more, the LIPE-AS1 level in CC cell lines was dramatically higher than that in normal cervical epithelial cells (Figure 1D). These results suggested that LIPE-AS1 expression is raised in cervical cancer and is a good predictor for poor prognosis.

**Figure 1:** LIPE-AS1 is increased in cervical cancer and related to worse survival. **(A,B)** LIPE-AS1 expression in 42 cases of cervical cancer tissues and the adjacent normal tissues were detected by RT-PCR, *P < 0.05, ***P < 0.001. **(C)** LIPE-AS1 expression in Cervical squamous cell carcinoma and endocervical adenocarcinoma (CESC) was analyzed through the GEPIA database (http://gepia.cancer-pku.cn/). **(D)** RT-PCR was taken to measure LIPE-AS1 expression in normal cervical epithelial cell lines HUCEC and cervical cancer cell lines (including Hela, MS751, SiHa, CaSki, C-33A, and HCC94). *P < 0.05, ***P < 0.001 vs. HUCEC group.

**Table 1:** Correlation between LIPE-AS1 expression and clinicopathological characteristics in cervical cancer patients.

		**LIPE-AS1 expression**		
**Characteristics**	**Cases**	**Low expression**	**High expression**	***P-*value**
**Age**				
<50	20	9	11	0.569
≥50	22	8	14	
**Tumor size (cm)**				
<4	26	11	15	0.758
≥4	16	6	10	
**Family history**				
Yes	19	9	10	0.408
No	23	8	15	
**FIGO stage**				
I–II	14	10	4	0.004
III	28	7	21	
**Lymph metastasis**				
Yes	15	10	5	0.010
No	27	7	20	

### LIPE-AS1 Promotes CC Cell Proliferation, Invasion, and EMT

To further investigate the effects of LIPE-AS1 on CC proliferation, apoptosis, invasion and EMT, a LIPE-AS1 overexpression or knockdown cell model was constructed in HCC94 and Hela cells, respectively (Figures 2A,B). The results of CCK-8 assay and BrdU assay illustrated that silencing LIPE-AS1 significantly reduced CC cell proliferation, while over-expressed LIPE-AS1 accelerated cell proliferation (Figures 2C–F). Besides, the apoptosis of cells was determined by flow cytometry, and the results showed that LIPE-AS1 overexpression led to lower apoptotic level while LIPE-AS1 knockdown enhanced cell apoptosis (Figures 2G,H). Transwell experiment showed that after overexpression of LIPE-AS1 in Hela cells, the invasive ability was considerably increased, while silencing LIPE-AS1 in HCC94 cells remarkably reduces their invasive ability (Figures 2I,J). What's more, western blot confirmed that over-expressed LIPE-AS1 significantly increased the protein expression of the mesenchymal markers (Vimentin and Snail), while decreased the protein level of the epithelial marker E-cadherin. However, silencing LIPE-AS1 produced the opposite results (Figure 2K). Hence, the above results revealed that LIPE-AS1 accelerates CC cell proliferation, invasion and EMT, and inhibits apoptosis.

**Figure 2:** LIPE-AS1 promotes cervical cancer cell proliferation, invasion, and EMT. LIPE-AS1 over- and low-expressing cell models were constructed in HeLa **(A)** and HCC94 cells **(B)**, respectively. CCK8 was applied to examine the proliferation of HeLa **(C)** and HCC94 cells **(D)**. *P < 0.05, **P < 0.01 vs. Vector group or sh-NC group. BrdU method was taken to examine the proliferation of HeLa **(E)** and HCC94 cells **(F)**. Flow cytometry was performed to test the apoptosis of HeLa **(G)** and HCC94 cells **(H)**. Transwell method was performed to evaluate the invasion of HeLa **(I)** and HCC94 cells **(J)**. **(K)** The expressions of E-cadherin, Snail and Vimentin in HeLa and HCC94 cells were detected by Western blot. *P < 0.05, **P < 0.01, ***P < 0.001. *N* = 3.

### LIPE-AS1 Targets miR-195-5p

For the purpose to verify the downstream target of LIPE-AS1, we browsed Starbase (http://starbase.sysu.edu.cn/) for searching the candidate targets of LIPE-AS1. It turned out that there are binding sites between LIPE-AS1 and miR-195-5p (Figure 3A). By detecting the level of miR-195-5p in CC tissues via RT-PCR, it was illustrated that miR-195-5p was drastically downregulated in CC tissues (compared with that of the normal tissues) (Figure 3B) and negatively correlated with LIPE-AS1 expression (Figure 3C). What's more, miR-195-5p displayed lower expression in many cancer types including CC (compared with normal tissues) (Figure 3D). Furthermore, the targeting relationship between LIPE-AS1 and miR-195-5p was clarified by dual luciferase activity experiment and RIP experiment. The data showed that miR-195-5p significantly inhibited luciferase activity of LIPE-AS1-WT, but had no obvious effect on LIPE-AS1-MUT (Figure 3E). RIP assay showed that higher level of LIPE-AS1 and miR-195-5p were enriched by anti-Ago2 antibody (compared with the IgG group) (Figure 3F). Furthermore, over-expressing LIPE-AS1 inhibited miR-195-5p expression while silencing LIPE-AS1 promoted miR-195-5p expression (Figures 3G–I). These results identified that miR-195-5p was the target molecule of LIPE-AS1, which may affect as a ceRNA.

**Figure 3:** LIPE-AS1 targets miR-195-5p. **(A)** Through browsing the Starbase database (http://starbase.sysu.edu.cn/), we analyzed the targeted miRNAs of LIPE-AS1 and found that miR-195-5p had complementary bases paired with LIPE-AS1. **(B,C)** The expression of miR-195-5p in cervical cancer tissues and adjacent normal tissues was measured by RT-PCR **(B)**, and the correlation between LIPE-AS1 and miR-195-5p in cervical cancer tissues was analyzed by linear regression. **(D)** miR-195-5p expression in human tumor tissues (data from the TCGA database). **(E)** The relationship between LIPE-AS1-miR-195-5p was verified via dual luciferase activity experiment. **(F)** The relationship between LIPE-AS1-miR-195-5p was verified by RIP experiments, and the enrichment level of LIPE-AS1 in cell lysate was detected via RT-PCR. ^NS^*P* > 0.05, ***P < 0.001. **(G)** RT-PCR was applied to determine miR-195-5p expression in normal cervical epithelial cell line HUCEC and cervical cancer cell lines (including Hela, MS751, SiHa, CaSki, C-33A, and HCC94). **P < 0.01, ***P < 0.001 vs. HUCEC group. **(H,I)** RT-PCR detected changes in miR-195-5p after silencing or overexpressing LIPE-AS1. ***P < 0.001. *N* = 3. The arrow shows that miR-195-5p is down-regulated in CESC (Cervical squamous cell carcinoma and endocervical adenocarcinoma) tissues compared with that in the normal tissues.

### The Function of LIPE-AS1/miR-195-5p Axis in CC Cells

To further explore the regulatory effect of LIPE-AS1/miR-195-5p axis on cervical cancer cells, miR-195-5p mimics and inhibitors were used to, respectively, construct miR-195-5p over-expressed and low-expressed cell lines. LIPE-AS1 overexpressed plasmids or sh-LIPE-AS1 were transfected into the cells to perform the compensation experiment (Figure 4A). The altered proliferation of HeLa and HCC94 cells were examined via CCK8 and BrdU methods. The results represented that miR-195-5p mimics suppressed HeLa cell proliferation, while the compensation of LIPE-AS1 over-expressed plasmids inhibited the effect of the miR-195-5p mimics. Besides, the miR-195-5p inhibitors promoted HCC94 cell proliferation, while compensation of sh-LIPE-AS1 inhibited the proliferation promotive effect of miR-195-5p inhibitors (Figures 4B,C). Then flow cytometry assay showed that miR-195-5p upregulation promoted cell apoptosis, and miR-195-5p downregulation reduced cell apoptosis (Figure 4D). What's more, results of transwell and western blot revealed that miR-195-5p mimic restrained CC cell invasion and EMT, while compensated LIPE-AS1 reversed the effects induced by miR-195-5p mimic (Figures 4E–G). Those data suggested that miR-195-5p exerted anti-tumor roles in CC. However, LIPE-AS1 overexpression markedly reversed miR-195-5p-mediated inhibitive effects in CC cells via enhancing cell proliferation, invasion, EMT and mitigating apoptosis (Figures 4B–G). Collectively, these experiments confirmed that miR-195-5p exerted a tumor inhibitive effects in CC, while LIPE-AS1 can marked those effect by targeting miR-195-5p.

**Figure 4:** The function of LIPE-AS1/miR-195-5p in cervical cancer cells. **(A)** MiR-195-5p mimics and inhibitors were taken to construct miR-195-5p over- and down-expressing cell lines, respectively, and further transfected with LIPE-AS1 over-expressed plasmids or sh-LIPE-AS1 to perform compensation experiments. CCK8 method **(B)** and BrdU method **(C)** were employed to detect HeLa and HCC94 cell proliferation. **(D)** Flow cytometry was performed to test the apoptosis of HeLa and HCC94 cells. **(E)** Transwell method was carried out to examine HeLa and HCC94 cell invasion. The expressions of E-cadherin, Snail, and Vimentin in HeLa **(F)** and HCC94 cells **(G)** were examined by Western blot. **P < 0.01, ***P < 0.001 vs. Vector or sh-NC group. ^&^*P* < 0.05, ^&&^*P* < 0.01, ^&&&^*P* < 0.001 vs. LIPE-AS1 group or sh-LIPE -AS1 group. *N* = 3.

### The Function of LIPE-AS1/miR-195-5p Axis in CC *in vivo*

*In vivo* experiments were conducted to further verify the regulatory effect of LIPE-AS1/miR-195-5p axis on CC. We transfected LIPE-AS1 over-expressing plasmids and/or miR-195-5p mimics into HeLa cells (Figure 5A) and sh-LIPE-AS1 and/or miR-195-5p inhibitors into HCC94 cells (Figure 5E). We found that LIPE-AS1 over-expression inhibited miR-195-5p, and LIPE-AS1 knockdown promoted miR-195-5p level (Figures 5A,E). Next, tumor volume and weight were calculated. It was found that LIPE-AS1 upregulation significantly promoted tumor growth (Figures 5B–D), while supplementing miR-195-5p mimics inhibited tumor growth (Figures 5B–D). What's more, downregulating LIPE-AS1 repressing tumor growth and inhibiting miR-195-5p promoted tumor growth (Figures 5F–H). Western blot was conducted to detect EMT markers in the tumor tissues. Similar to the *in-vitro* data, LIPE-AS1 overexpression enhanced Snail and Vimentin level, reduced E-cadherin expression. After supplementing miR-195-5p mimics, Snail and Vimentin levels were reduced, and E-cadherin expression was enhanced (Figure 5I). On the other hand, downregulation of LIPE-AS1 led to reduced EMT and miR-195-5p inhibitors promoted EMT of CC cells *in vivo* (Figure 5J). The above results confirmed that LIPE-AS1 promoted tumor development *in vivo*, while miR-195-5p inhibited the oncogenic effects of LIPE-AS1.

**Figure 5:** The function of LIPE-AS1/miR-195-5p in cervical cancer cells *in vivo*. LIPE-AS1 plasmid or sh-LIPE-AS1 were used to construct cell models of LIPE-AS1 overexpression and knockdown, respectively, and further transfected with miR-195-5p mimic or inhibitor. The nude mouse tumor formation model was constructed with stably transfected cells. The expressions of LIPE-AS1 and miR-195-5p in HeLa cells **(A)** and HCC94 cells **(E)** were examined by RT-PCR, respectively. **(B,F)** Nude mice were sacrificed in the fifth week, and tumor tissue was removed. **(C,G)** Tumor volume in nude mice; **(D,H)** tumor mass at the fifth week; **(I,J)** western blot was taken to determine the expressions of E-cadherin, Snail, and Vimentin in tumor tissues. ^NS^*P* > 0.05, *P < 0.05, **P < 0.01, ***P < 0.001. ^&^*P* < 0.05, ^&&^*P* < 0.01, ^&&&^*P* < 0.001 vs. LIPE-AS1 group or sh-LIPE-AS1 group. *N* = 4.

### MiR-195-5p Targets MAP3K8

For the purpose to identify the underlying mechanisms of the miR-195-5p in regulating CC development, we performed bioinformatics analysis through mirPath v.3 (http://snf-515788.vm.okeanos.grnet.gr/index.php?r=mirpath). There were 62 related pathways regulated by miR-28-5p including cervical cancer (Figure 6A). Then, we conducted bioinformatics analysis through miRmap (http://mirnamap.mbc.nctu.edu.tw/), MicroT (https://omictools.com/diana-microt-cds-tool), and Targetscan (http://www.targetscan.org/vert_72/) to predict miR-195-5p targeting genes (Figure 6B) and Venn diagram was used to analyze the co-targets regulated by miR-195-5p in those databases. The results showed that 15 candidate genes were selected (Figure 6C). Next, we employed qRT-PCR to evaluate the 15 candidate genes in cervical cancer cells transfected with miR-195-5p mimics. The statistics indicated that miR-195-5p significantly decreased MAP3K8 expression (Figure 6D). Meanwhile, MAP3K8 was found to be a direct candidate target of miR-195-5p in starbase (http://starbase.sysu.edu.cn/index.php) (Figure 6E). Basing on those data, we carried out dual luciferase reporter gene assay. It was found that miR-195-5p targeted on the 3'UTR sites of MAP3K8 (Figure 6F). Moreover, the western blot and cell immunofluorescence results revealed that over-expressing miR-195-5p considerably decreased the MAP3K8 on protein level (Figures 6G,H). Thus, those data demonstrated that miR-195-5p had significant effect on MAP3K8 pathway modulation.

**Figure 6:** MiR-195-5p targets MAP3K8. **(A)** The mirpath database (http://snf-515788.vm.okeanos.grnet.gr/index.php?r=mirpath) was used to predict the signal pathways regulated by miR-195-5p. **(B)** Through mirmap (http://mirnamap.mbc.nctu.edu.tw/), microT (https://omictools.com/diana-microt-cds-tool), and Targetscan (http://www.targetscan.org/vert_72/), miR-195-5p's targeting molecule was predicted. **(C)** The miR-195-5p related molecules in mirpath, mirmap, microT, and Targetscan databases were analyzed by Venn diagram. **(D)** RT-PCR was performed to measure tumor gene expression after miR-195-5p overexpression. **(E)** Base pairing between miR-195-5p and MAPK8. **(F)** Dual luciferase activity experiments were applied to verify the relationship between miR-195-5p and MAPK8. **(G)** Western blot was taken to evaluate the protein level of MAP3K8 in over-expressing miR-195-5p and low-expressing miR-195-5p cells. **(H)** Cell immunofluorescence was taken to evaluate the protein level of MAP3K8 in over-expressing miR-195-5p and low-expressing miR-195-5p cells. ^NS^*P* > 0.05, ***P < 0.001. *N* = 3.

### The Function of LIPE-AS1/miR-195-5p in MAPK/ERK Pathway

The effect of LIPE-AS1/miR-195-5p on the MAPK/ERK pathway was determined via western blot. It showed that the protein expressions of MAP3K8 and p-ERK were considerably increased in by overexpressing LIPE-AS1 (Figure 7A) but decreased by downregulating LIPE-AS1 (Figure 7B). Additionally, transfection of miR-195-5p mimics reduced protein levels of MAP3K8 and p-ERK in LIPE-AS1 overexpressed cells and transfection of miR-195-5p inhibitors obviously increased the protein expressions of MAP3K8 and p-ERK (Figures 7C,D). Furthermore, tissue immunofluorescence was performed to detect MAP3K8 expression in the tumor tissues. We found that LIPE-AS1 overexpression enhanced MAP3K8 expression while downregulating LIPE-AS1 suppressed MAP3K8 level. On the contrary, miR-195-5p mimics reduced MAP3K8 level in LIPE-AS1-overexoressed cells (Figures 7E,F). Therefore, the above data revealed that LIPE-AS1 regulates the MAPK/ERK pathway by sponging miR-195-5p (Figure 8).

**Figure 7:** The effect of LIPE-AS1/miR-195-5p on the MAPK/ERK pathway. LIPE-AS1 over- and low-expressing cell models were constructed in HeLa **(A)** and HCC94 cells **(B)**, respectively. Western blot was used to measure MAP3K8 and ERK protein expression in the cells. **(C,D)** Transfection of cervical cancer cells with miR-195-5p mimics and inhibitors, LIPE-AS1 over-expressed plasmid or sh-LIPE-AS1. Western blot was taken to measure the protein expressions of MAP3K8 and ERK in cells. **(E,F)** Tissue immunofluorescence was carried out to detect MAP3K8 in the tumor tissues (the grouping was the same as Figure 5). *P < 0.05, **P < 0.01, ***P < 0.001. *N* = 3.

**Figure 8:** The mechanism diagram. During the progression of cervical cancer (CC), LIPE-AS1 is upregulated and inhibits the expression of miR-195-5p, which targets at the 3′UTR of MAP3K8 mRNA. Low level of miR-195-5p leads to overexpressed MAP3K8 thus enhancing the phosphorylation of ERK. The activation of MAPK/ERK pathway increases the proliferation, viability, invasion, and EMT of CC cells, therefore promoting the development of CC.

## Discussion

Along with the unceasing thorough researches on CC, mounting lncRNAs have been found to participate in cervical cancer occurrence and progression. Hence, the study of the biological function and potential mechanism of lncRNA in cervical cancer is very important for the exploration of new therapeutic targets for cervical cancer. Here, LIPE-AS1 expression was found remarkably up-regulated in CC and it also accelerated CC development by regulating miR-195-5p /MAPK pathway.

The effects of lncRNAs on cancers has been a research focus. What's more, a large number of papers have stated that lncRNA exerts an important regulatory effect on CC. For example, lncRNA MIR210HG (4), CCAT1 (5), FOXD2-AS1 (14), DLX6-AS1 (15), BLACAT1 (16), and other lncRNSs have been reported to promote cervical cancer development. However, lncRNAs such as PTENP1 (6) and WT1-AS (17), etc. have been reported to inhibit CC progression. Hence, different lncRNAs may play different roles in CC development. Although there have been few reports on the effect of LIPE-AS1 in cancer, only Goyal et al. has reported that LIPE-AS1 is associated with DNA damage in cancer cells (7). However, through database analysis and studies on CC tissues and cells (Figure 1), it was found that LIPE-AS1 expression in CC was significantly increased with high expression abundance. Therefore, the present study initially investigated the role and mechanism of LIPE-AS1 in CC. The experiment results illustrated that LIPE-AS1 notably promotes CC proliferation, invasion and tumor formation, suggesting that LIPE-AS1 is a promising therapeutic target for CC.

Recently, it has been reported that miRNAs make great contributions in CC development. More importantly, miR-195-5p, as a relatively common type of miRNA, plays an inhibitory role in a variety of tumors. For instance, miR-195-5p has been reported to restrain the malignant biological behaviors of tumors such as non-small cell lung lancer (18), osteosarcoma (19), and thyroid cancer (20). Besides, several studies also indicate that miR-195-5p inhibits CC cell proliferation and invasion through various mechanisms (8, 9). In CC, lncRNA exerts its effect by sponging miRNA (21). However, whether LIPE-AS1 could target miR-195-5p has not been reported. This study confirmed that miR-195-5p exerts an inhibitive effect in CC by restraining the proliferation, invasion and EMT of CC cells. More importantly, the study here initially clarified that LIPE-AS1 exerts a regulatory effect on CC by sponging miR-195-5p.

For further research on the downstream mechanism, we screened out MAP3K8 as a candidate target of miR-195-5p (Figure 6). MAP3K8 (mitogen2 activated protein kinase 8) gene, also known as JNK1/ SAPK1 gene, is an important signaling molecule in the signal transduction pathway of MAPK, whose functions are involved in various mechanisms such as cell proliferation, differentiation and apoptosis (22). In addition, numerous studies have proved that MAP3K8 activates the downstream ERK signaling pathway which promotes tumor development, especially in melanoma. In addition, abundant literatures have identified the effect of multiple miRNAs in tumor inhibition by targeting MAP3K8. Zhang et al. reported that miR-589-5p overexpression inhibited the stem cell characteristics of CD90 cells and functioned by targeting MAP3K8, which provided a new molecular target for HCC treatment (12). What's more important, microRNA-375 may inhibit the expression of the downstream gene ERK in tumor tissues by targeting MAP3K8, thus inhibiting the proliferation of colon cancer cells and notably reducing tumor formation in nude mice (23). However, the regulatory effect of miR-195-5p in the regulation of MAP3K8 in tumors has not been reported. Only Akama et al. reported that miR-195 overexpression inhibited TSH-induced cell cycle progression and DNA synthesis, possibly by targeting MAP3K8 (24, 25). Considering the anti-tumor effect of miR-195-5p in many tumors and its close relationship with MAP3K8 confirmed by the TCGA database (Figure 6), it is indicated that miR-195-5p may inhibit CC by targeting MAPK8/ERK. These experimental results further confirmed the above hypothesis.

In conclusion, our results indicate that LIPE-AS1 expression in CC tissues and cells is significantly up-regulated and is involved in CC development by regulating the ERK signaling pathway mediated by miR-195-5p /MAP3K8 axis (Figure 8). This study may provide a meaningful basis for a more profound understanding of the biological behavior of LIPE-AS1 in CC, as well as for the early diagnosis and treatment of CC.

## Data Availability Statement

The datasets presented in this study can be found in online repositories. The names of the repository/repositories and accession number(s) can be found in the article/Supplementary Material.

## Ethics Statement

The studies involving human participants were reviewed and approved by the Ethics Review Board of the First Affiliated Hospital of Nanjing Medical University. The patients/participants provided their written informed consent to participate in this study.

## Author Contributions

SF and WC: conceived and designed the experiments. JZ and PJ: performed the experiments and wrote the paper. SW: statistical analysis. All authors read and approved the final manuscript.

## Conflict of Interest

The authors declare that the research was conducted in the absence of any commercial or financial relationships that could be construed as a potential conflict of interest.
